The article "VGLL4 Protects against Oxidized-LDL-Induced Endothelial Cell Dysfunction and Inflammation by Activating Hippo-YAP/TEAD1 Signaling Pathway" was retracted in 2022. Reasons: manipulated images; duplicated images.

# VGLL4 Protects against Oxidized-LDL-Induced Endothelial Cell Dysfunction and Inflammation by Activating Hippo-YAP/TEAD1 Signaling Pathway

**DOI:** 10.1155/2020/8292173

**Published:** 2020-12-30

**Authors:** Kaicheng Xu, Haomin Zhao, Xiaolei Qiu, Xiwen Liu, Fucheng Zhao, Yue Zhao

**Affiliations:** ^1^Department of Anesthesiology, China-Japan Union Hospital, Jilin University, Changchun, Jilin 130033, China; ^2^Department of Vascular Surgery, China-Japan Union Hospital, Jilin University, Changchun, Jilin 130033, China

## Abstract

Vestigial-like 4 (VGLL4) has been found to have multiple functions in tumor development; however, its role in cardiovascular disease is unknown. The aim of this study was to investigate the effect of VGLL4 on the dysfunction and inflammatory response of Ox-LDL-induced human umbilical vein endothelial cells (HUVECs) and its mechanism, so as to provide a new theoretical basis for the diagnosis and treatment of atherosclerosis. In the present study, the protective activity of VGLL4 inhibiting Ox-LDL-induced apoptosis, oxidative stress, inflammation, and injury as well as its molecular mechanisms was examined using human umbilical vein endothelial cells (HUVECs). The results showed that the expression of VGLL4 was decreased with the increase of Ox-LDL concentration in HUVECs. In addition, the functional study found that VGLL4 overexpression alleviated Ox-LDL-induced oxidative stress, inflammation, and dysfunction and inhibited apoptosis. Further research found that VGLL4 regulated Hippo-YAP/TEAD1 signaling pathway, and the Hippo-YAP/TEAD1 signaling pathway was involved in the protective mechanism of VGLL4 on HUVECs. In conclusion, it suggests that VGLL4 protects against oxidized-LDL-induced endothelial cell dysfunction by activating the Hippo-YAP/TEAD1 signaling pathway.

## 1. Introduction

Atherosclerosis (AS) is the most common cardiovascular disease, which is a slow progressive disease [1]. The involved artery lesions begin from the intima, and there is lipid accumulation, fibrous tissue hyperplasia, and calcium deposition in the local area, forming plaques [2]. According to the statistics, about 20 million people die of atherosclerosis every year in the world [3]. With the continuous development of modern medical drug treatment, surgical treatment, interventional treatment, and other methods, the mortality rate of atherosclerosis is showing a downward trend, but the incidence is still increasing [4].

Vestigial-like 4 (VGLL4) is an important member of the vascular like protein (VGLL) family [5]. VGLL is a new kind of protein which is involved in tumor development in recent years. There are four members of VGLL proteins in mammals, named VGLL1-4 [6]. Previous studies have shown that VGLL1 promotes cell proliferation and is highly expressed in basal breast cancer [7]. Similarly, VGLL3 is amplified in soft tissue sarcoma, and the inhibition of VGLL3 results in the decrease of cell proliferation and migration [8]. Unlike other members of the VGLL family, VGLL4 contains an additional TDU domain and is considered functionally different [9]. However, the role of VGLL4 in the development of cardiovascular disease needs to be further explored.

The article "VGLL4 Protects against Oxidized-LDL-Induced Endothelial Cell Dysfunction and Inflammation by Activating Hippo-YAP/TEAD1 Signaling Pathway" was retracted in 2022. Reasons: manipulated images; duplicated images.

The Hippo signaling pathway is a highly conserved growth control signaling pathway [10]. It was initially found in Drosophila cells that inhibit cell proliferation and induce cell apoptosis, play an important role in the process of embryonic development, tissue, and organ formation, and also have a direct relationship with the occurrence and development of tumors [11]. Yap, a multifunctional intracellular connexin and transcription coactivator, plays a central role in the Hippo signaling pathway. At present, the study of Hippo/Yap signaling pathway is more limited in tumor, but in recent years, there are more and more reports about its role in cardiovascular disease [12]. Related studies show that the Hippo/Yap signaling pathway plays an important role in cardiovascular development, hypertrophy, apoptosis, autophagy, angiogenesis, and regeneration [13]. However, the role of the Hippo signaling pathway in the development of AD has not been fully elucidated, which needs to be further explored. In addition, VGLL4 can regulate the activation of the Hippo signaling pathway. For example, VGLL4 regulates the Hippo-Yap/TEAD signal pathway during cardiac development. VGLL4 not only regulates the stability of TEAD but also regulates its interaction with Yap [14]. Therefore, this study will explore the role of VGLL4/Hippo-Yap/TEAD axis in atherosclerosis.

In the present study, we explored the effect of VGLL4 on the dysfunction of HUVECs and the special molecular mechanism. Our results demonstrated that VGLL4 protects against oxidized-LDL-induced endothelial cell dysfunction by activating the Hippo-YAP/TEAD1 signaling pathway. It is suggested that VGLL4 may be a potential target for the treatment of cardiovascular disease.

## 2. Materials and Methods

### 2.1. Cell Culture

The HUVECs were cultured at 37°C with 5% CO_2_. The medium components used include 10% fetal bovine serum (EBM-2, Lonza) (Solarbio, Beijing, China), 1% glutamine (Invitrogen, Carlsbad, CA, USA), 100 U/mL penicillin sodium, and 100 *μ*g/mL streptomycin sulfate (Invitrogen, Carlsbad, CA, USA).

### 2.2. Reagents

The materials used are as follows: the HUVECs (San Diego, CA, USA); GAPDH, anti-VGLL4 (1 : 2000), anti-VCAM-1(1 : 2000), anti-TEAD1 (1 : 500), anti-YAP (1 : 500), anti-caspase-3 (1 : 1000), anti-caspase-9 (1 : 500), and anti-ICAM-1 (1 : 1000) (Beijing TsingKe Biotechnology Co., Ltd., Beijing, China); DMEM (Beyotime Biotechnology, China); WST-8 (Solarbio, Beijing, China); RNA extraction kits, RT-PCR kits (Beyotime Biotechnology, China), reverse transcription kits, ELISA kits (Westang Technology Ltd., Shanghai, China); and primer synthesis (Beijing TsingKe Biotechnology Co., Ltd., Beijing, China). The sequences of primers used in the present study are presented in Table 1.

The article "VGLL4 Protects against Oxidized-LDL-Induced Endothelial Cell Dysfunction and Inflammation by Activating Hippo-YAP/TEAD1 Signaling Pathway" was retracted in 2022. Reasons: manipulated images; duplicated images.

### 2.3. Plasmids

The overexpression vector of VGLL4 was constructed according to the literature. In this study, all plasmids were constructed in the modified pcDNA3.1 vector. The VGLL4 sequences were cloned into the plasmid pcDNA3.1 using PCR. The pcDNA3.1 without the VGLL4 genes was a negative control (2 *μ*g/mL). pcDNA3.1-VGLL4 was transfected into the HUVECs (6-well plate, 1.0 × 10^5^/cm^2^).

### 2.4. Transfection

pcDNA3.1-VGLL4, si-YAP, si-TEAD, and Ctrl-siRNA were designed and synthesized by Tsingke Biotech Co., Ltd. (Beijing, China). The HUVECs were inoculated into 6-well plate with a density of 1 × 10^6^ cells/well. Transfection assay was performed according to the instructions of cell transfection kit (Solarbio, Beijing, China).

### 2.5. CCK-8 Assay

The HUVECs were inoculated into 96-well plate and cultured in 37°C for 24 h. 2-(2-Methoxy-4-nitrophenyl)-3-(4-nitrophenyl)-5-(2,4-disulfobenzene (WST-8) (10 *μ*L) was added to the plate well for 24 h. Optical density (OD) value at 450 nm was determined by microplate reader.

### 2.6. ELISA Assay

The concentrations of TNF-*α* and IL-6 in the supernatants were detected using the corresponding ELISA kits (Westang Technology Ltd., Shanghai, China) according to the instructions.

### 2.7. Annexin V-FITC/PI

The HUVECs were inoculated into 6-well plates for 24 h. Apoptosis experiments in this study were detected using the corresponding Annexin V-FITC apoptosis detection kits (Solarbio, Beijing, China) according to the instructions. We followed the methods of Xu et al. [15].

### 2.8. Measurement of ROS

The HUVECs were incubated into 6-well plates overnight. The cells were collected and incubation with ROS indicator DCFH-DA (20 *μ*M) in PBS for 30 min at 37°C. The fluorescence was analyzed using fluorescence microscope (BD Biosciences, CA) and fluorescence microplate reader. We followed the methods of Xu et al. [15].

### 2.9. Measurement of NAD^+^

Intracellular NAD^+^ levels were measured using the EnzyChrom NAD^+^/NADH assay kit (BioAssay Systems, Hayward, CA, U.S.A.). The HUVECs were washed with PBS and then lysed with the supplied NAD extraction buffer. NAD^+^ was extracted from the lysate according to the manufacturer's protocol. The measurement of NAD^+^ is based on an alcohol dehydrogenase cycling reaction. The change in absorbance at 565 nm for 15 min at room temperature was measured.

The article "VGLL4 Protects against Oxidized-LDL-Induced Endothelial Cell Dysfunction and Inflammation by Activating Hippo-YAP/TEAD1 Signaling Pathway" was retracted in 2022. Reasons: manipulated images; duplicated images.

### 2.10. Measurement of ATP

The HUVECs were treated with the culture medium and replaced by HEPES buffer. After washing, the initially stored culture medium was added to cells for 1 h. The cells were lysed with 10 mM Tris-HCl (pH 7.8), and the ATP content was determined using a quantitative bioluminescent assay (Sigma, St. Louis, MO, U.S.A.) according to the instructions of the manufacturer and an iMark microplate absorbance reader (Bio-Rad, Hercules, CA, USA).

### 2.11. RT-qPCR

Total RNA samples from the HUVECs were isolated using TRIzol® reagent (Solarbio, Beijing, China), and the RNA concentration was measured by Nanodrop 2000. Then, the total RNA was retrotranscribed into cDNA according to the instructions of the reverse transcription kits. According to the instructions of qPCR kits, we configure the corresponding system and set up 3 multiple wells for each group. The conditions of qPCR were as follows: 95°C 1 min (1 cycle), 95°C 20 s, 60°C 1 min (32 cycles). The data were analyzed by the 2^–*ΔΔ*CT^ method with GAPDH as a normalizing gene. We followed the methods of Xu et al. [15].

### 2.12. Western Blotting

The HUVECs were seeded in a 6-well plate at a density of 1 × 10^5^ cells/well. The HUVECs were lysed with improved RIPA buffer (Solarbio, Beijing, China). The extracted protein (30 *μ*g) was separated from denatured polyacrylamide gel and then transferred to PVDF membrane, sealed with 5% skim milk (Solarbio, Beijing, China). Then, the enhanced laboratories (ECL) darkroom development, Bio-Rad Laboratories (California, USA) scan record, and anti-GAPDH as internal reference were used for analysis and comparison. We followed the methods of Xu et al. [15].

### 2.13. Statistical Analyses

All the data were presented as mean + SD, and each experiment were performed in triplicate. One-way ANOVA was used to analyze statistical significance. All statistical analyses were performed by the SPSS 20.0 software (SPSS, Inc., Chicago, IL, USA). *P* value < 0.05 was considered significant.

## 3. Results

### 3.1. The Expression of VGLL4 Is Lower in Ox-LDL-Induced HUVECs

The HUVECs were treated with Ox-LDL (25, 50, 100, and 200 *μ*g/mL). As shown in Figure 1(a), cell viability of HUVECs was significantly decreased by Ox-LDL induced in a dose-dependent manner (Figure 1(a)). What is more, the mRNA expression of VGLL4 was decreased in Ox-LDL-treated HUVECs (Figure 1(b)). As expected, the protein expression of VGLL4 was also significantly downregulated in HUVECs (Figure 1(c)).

The article "VGLL4 Protects against Oxidized-LDL-Induced Endothelial Cell Dysfunction and Inflammation by Activating Hippo-YAP/TEAD1 Signaling Pathway" was retracted in 2022. Reasons: manipulated images; duplicated images.

### 3.2. Overexpression of VGLL4 Alleviates Ox-LDL-Induced Oxidative Stress and Inflammation in HUVECs

The HUVECs were transfected with the pcDNA3.1 (pcDNA3.1 group) or pcDNA3.1-VGLL4 (p-VGLL4 group), respectively. After pcDNA3.1-VGLL4 being transfected, the expression of VGLL4 protein significantly increased (Figure 2(a)). In addition, overexpression of VGLL4 alleviates Ox-LDL-induced oxidative stress. As shown in Figures 2(b)–2(d), VGLL4 significantly decreased the ROS level of Ox-LDL-induced HUVECs, while significantly increased the ATP and NAD^+^ level (Figures 2(b)–2(d)). As expected, the levels of IL-6 and TNF-*α* were significantly increased after Ox-LDL treatment, while pcDNA3.1-VGLL4 significantly downregulated the expression of IL-6 and TNF-*α* (Figures 2(e) and 2(f)).

### 3.3. Overexpression of VGLL4 Inhibits Ox-LDL-Induced Apoptosis in HUVECs

As shown in Figure 3(a), Ox-LDL significantly decreased the cell viability of HUVECs, while pcDNA3.1-VGLL4 significantly reversed the inhibited effect of Ox-LDL (Figure 3(a)). In addition, the apoptosis rate of HUVECs was increased after Ox-LDL treatment compared with the untreated group, while overexpression of VGLL4 alleviates Ox-LDL-induced apoptosis (Figure 3(b)). As expected, the protein expression of caspase-3 and caspase-9 was significantly increased in the Ox-LDL treatment group, while pcDNA3.1-VGLL4 significantly decreased the expression of caspase-3 and caspase-9 (Figure 3(c)).

### 3.4. Overexpression of VGLL4 Alleviates Ox-LDL-Induced Dysfunction in HUVECs

VCAM-1, ICAM-1, and MCP-1 are important adhesion factors that affect the occurrence and development of cardiovascular diseases [16]. The protein expression of VCAM-1, ICAM-1, and MCP-1 was significantly increased after Ox-LDL treatment. In contrast, VGLL4 significantly downregulated the expression of VCAM-1, ICAM-1, and MCP-1 in HUVECs (Figures 4(a)–4(d)). As expected, the protein expression of iNOS was significantly increased in Ox-LDL treatment group, while pcDNA3.1-VGLL4 significantly decreased the expression of iNOS, while the expression of eNOS showed an opposite trend (Figure 4(e)).

### 3.5. Overexpression of VGLL4 Promotes the Expression of YAP and TEAD1, and Ox-LDL Inhibits the Expression of YAP and TEAD1

The protein expression YAP and TEAD1 was significantly increased in the pcDNA3.1-VGLL4 group compared with the control group and pcDNA3.1 group (Figure 5(a)). In addition, the protein expression of YAP and TEAD1 was decreased in Ox-LDL-treated HUVECs in a dose-dependent manner (Figure 5(b)).

### 3.6. Hippo-YAP/TEAD1 Signaling Pathway Is Involved in the Protective Mechanism of VGLL4 on HUVECs

The results showed that si-YAP and si-TEAD1 significantly decreased the cell viability of HUVECs (Figure 6(a)). In addition, pcDNA3.1-VGLL4 significantly decreased the apoptosis rate of HUVECs, while si-YAP and si-TEAD1 reversed the inhibited effect of VGLL4 (Figure 6(b)). Furthermore, the production of ROS was significantly reduced after being transfected with pcDNA3.1-VGLL4. In contrast, si-YAP and si-TEAD1 reversed the inhibited effect of VGLL4 on production of ROS (Figure 6(c)). As shown in Figure 6(d), the level of IL-6 was increased after si-YAP and si-TEAD1 treatment compared with the control group in HUVECs (Figure 6(d)). What is more, si-YAP and si-TEAD1 increased the protein expression of VCAM-1, and reversed the inhibited effect of VGLL4 (Figure 6(e)).

The article "VGLL4 Protects against Oxidized-LDL-Induced Endothelial Cell Dysfunction and Inflammation by Activating Hippo-YAP/TEAD1 Signaling Pathway" was retracted in 2022. Reasons: manipulated images; duplicated images.

## 4. Discussion

Studies have shown that the HUVECs have been used in many cardiovascular disease models, including hypertension, hyperlipidemia, coronary heart disease, and atherosclerosis. In addition, Ox-LDL-induced HUVECs model is one of the commonly used models in the study of atherosclerosis. Our previous studies have shown that Ox-LDL-treatment promotes inflammation and dysfunction of HUVECs [15]. Similarly, the present research has reached a consistent conclusion. In this study, we found that VGLL4 alleviated Ox-LDL-induced oxidative stress, inflammation, and dysfunction and inhibited apoptosis in HUVECs. Furthermore, the Hippo-YAP/TEAD1 signaling pathway is involved in the protective mechanism of VGLL4 on HUVECs. Therefore, VGLL4 may be a new target for cardiovascular disease.

Previous studies have shown that VGLL4, as a tumor suppressor, plays a key role in the development of a variety of tumors [5, 6, 17]. However, its role in cardiovascular system has not been elucidated. It is necessary to further explore the role and mechanism of VGLL4 in atherosclerosis, so as to provide a new theoretical basis for the diagnosis and treatment of atherosclerosis. Therefore, the purpose of this study is to explore the role of VGLL4 in the development of atherosclerosis and its molecular mechanism. In this study, VGLL4 was found to protect HUVECs from inflammation and injury. Interestingly, Jin et al. [18] reported that VGLL4, by combining with inhibition of apoptotic protein (IAP), inhibits cardiomyocyte apoptosis and participates in the development of the heart, thus protecting the biological function of heart development. Coincidentally, acetylated VGLL4 regulates the cardiac development of neonates by regulating the YAP/TEAD1 signal pathway [14]. Consistent with this, we found that VGLL4 regulated the expression of key proteins in Hippo-YAP/TEAD1 signaling pathway, including TEAD1 and YAP, to further alleviate the development of atherosclerosis. However, VGLL4 may play a biological role in the pathogenesis of atherosclerosis by regulating other signaling pathways. As we all know, YAP/TEAD1 is closely related to Wnt/*β*-catenin, so next, we will investigate the regulation of VGLL4 on the Wnt/*β*-catenin signaling pathway.

The article "VGLL4 Protects against Oxidized-LDL-Induced Endothelial Cell Dysfunction and Inflammation by Activating Hippo-YAP/TEAD1 Signaling Pathway" was retracted in 2022. Reasons: manipulated images; duplicated images.

At present, there are still disputes about the mechanism of VGLL4 regulating the Hippo-YAP/TEAD1 signaling pathway [5, 19, 20]. Previous studies have shown that VGLL4 inhibits YAP activity by competing for the binding of VGLL4 [21, 22]. While Lin et al. have found another special regulatory mechanism. They found that VGLL4 combined with TEAD1 accelerated the degradation of TEAD1 by cysteine peptidase. The results showed that VGLL4 regulated the activity of YAP-TEAD1 by inducing the degradation of TEAD1 and inhibiting the interaction of YAP-TEAD1 [14]. Therefore, the regulation mechanism of VGLL4 on the Hippo-YAP/TEAD1 signaling pathway needs to be further explored.

The occurrence of diseases is often related to the dysfunction of key signaling pathways, such as the Hippo-YAP signaling pathway [23, 24]. As we all know, the Hippo-YAP signaling pathway plays an important role in the development of the heart and participates in various physiological and pathological processes, including cardiovascular development, cardiac hypertrophy, angiogenesis, and regeneration [25–27]. Healen et al. have confirmed that cardiac-specific knockout of SAV1 can block the Hippo-YAP/TEAD1 signaling pathway, significantly reduce the level of Yap phosphorylation, and lead to cardiac hypertrophy, which has also been verified in MST1/2 and LATS2 knockout mice [28–30]. In addition, the Hippo-YAP/TEAD1 signaling pathway is closely related to cardiovascular disease including atherosclerosis. It is reported that Hippo-Yap, as a target of traditional Chinese medicine, protected endothelial cells from injury and inhibited apoptosis to slow down the process of atherosclerosis [31]. Coincidentally, we found that the Hippo-YAP/TEAD1 signaling pathway was involved in the protective mechanism of VGLL4 on HUVECs. It can be inferred that the Hippo-YAP/TEAD1 signaling pathway may be widely participated in the regulatory network of cardiovascular disease.

In conclusion, we explored the protect effect of VGLL4 on the process of AS and the special molecular mechanism. We found that VGLL4 alleviated the Ox-LDL-induced oxidative stress, inflammation, and dysfunction via regulating the Hippo-YAP/TEAD1 signaling pathway. It suggests that VGLL4 may be a potential target for the treatment of AS.

The article "VGLL4 Protects against Oxidized-LDL-Induced Endothelial Cell Dysfunction and Inflammation by Activating Hippo-YAP/TEAD1 Signaling Pathway" was retracted in 2022. Reasons: manipulated images; duplicated images.

## Figures and Tables

**Figure 1:** The expression of VGLL4 is lower in Ox-LDL-induced HUVECs. (a) The CCK-8 was used to detect cell viability of HUVECs. (b) The mRNA expression of VGLL4 in HUVECs treated with Ox-LDL at 25, 50, 100, and 200 *μ*g/mL. (c) The protein expression of VGLL4 in HUVECs cells treated with Ox-LDL at 25, 50, 100, and 200 *μ*g/mL. “∗” means compared with the control group at *P* < 0.05. GAPDH was used as an invariant internal control for calculating protein fold changes.

**Figure 2:** Overexpression of VGLL4 alleviates Ox-LDL-induced oxidative stress and inflammation in HUVECs. The HUVECs were treated with Ox-LDL (100 *μ*g/mL) and transfected with the control vector (pcDNA3.1 group) or pcDNA3.1-VGLL4 (p-VGLL4 group), respectively. (a) The protein expression of VGLL4 in the untreated, control, pcDNA3.1, and p-VGLL4 groups. (b) The ROS level in the untreated, control, pcDNA3.1, and p-VGLL4 groups. (c) The NAD^+^ level in the untreated, control, pcDNA3.1, and p-VGLL4 groups. (d) The ATP level in the untreated, control, pcDNA3.1, and p-VGLL4 groups. (e) The IL-6 level in the untreated, control, pcDNA3.1, and p-VGLL4 groups. (f) The TNF-*α* level in the untreated, control, pcDNA3.1, and p-VGLL4 groups. “∗” means compared with the untreated group at *P* < 0.05, and “#” means compared with the pcDNA3.1 group at *P* < 0.05. GAPDH was used as an invariant internal control for calculating protein fold changes.

**Figure 3:** Overexpression of VGLL4 inhibits Ox-LDL-induced apoptosis in HUVECs. The HUVECs were treated with Ox-LDL (100 *μ*g/mL), and transfected with the control vector (pcDNA3.1 group) or pcDNA3.1-VGLL4 (p-VGLL4 group), respectively. (a) The cell viability in the untreated, control, pcDNA3.1, and p-VGLL4 groups. (b) The apoptosis of HUVECs in the untreated, control, pcDNA3.1, and p-VGLL4 groups. (c) The protein expression of caspase-3 and caspase-9 in the untreated, control, pcDNA3.1, and p-VGLL4 groups. “∗” means compared with the untreated group at *P* < 0.05, and “#” means compared with the pcDNA3.1 group at *P* < 0.05. GAPDH was used as an invariant internal control for calculating protein fold changes.

**Figure 4:** Overexpression of VGLL4 alleviates Ox-LDL-induced dysfunction in HUVECs. The HUVECs were treated with Ox-LDL (100 *μ*g/mL) and transfected with the control vector (pcDNA3.1 group) or pcDNA3.1-VGLL4 (p-VGLL4 group), respectively. (a) Western blot was performed to confirm the protein expression levels of VCAM-1, ICAM-1, MCP-1, iNOS, and eNOS. (b–d) The protein expression of VCAM-1, ICAM-1, and MCP-1 in the untreated, control, pcDNA3.1, and p-VGLL4 groups. (e) The protein expression of NOS and eNOS in the untreated, control, pcDNA3.1, and p-VGLL4 groups. “∗” means compared with the untreated group at *P* < 0.05, and “#” means compared with the pcDNA3.1 group at *P* < 0.05. GAPDH was used as an invariant internal control for calculating protein fold changes.

The article "VGLL4 Protects against Oxidized-LDL-Induced Endothelial Cell Dysfunction and Inflammation by Activating Hippo-YAP/TEAD1 Signaling Pathway" was retracted in 2022. Reasons: manipulated images; duplicated images.

**Figure 5:** Overexpression of VGLL4 promotes the expression of TEAD1 and YAP, and Ox-LDL inhibits the expression of TEAD1 and YAP. (a) The protein expression of TEAD1 and YAP in the control, pcDNA3.1, and p-VGLL4 groups. (b) The protein expression of TEAD1 and YAP in HUVECs cells treated with Ox-LDL at 25, 50, 100, and 200 *μ*g/mL. “∗” means compared with the untreated group at *P* < 0.05, and “#” means compared with the pcDNA3.1 group at *P* < 0.05. GAPDH was used as an invariant internal control for calculating protein fold changes.

**Figure 6:** The Hippo YAP/TEAD1 signaling pathway is involved in the protective mechanism of VGLL4 on HUVECs. The HUVECs were treated with Ox-LDL (100 *μ*g/mL) for 24 h and transfected with pcDNA3.1-VGLL4, si-TEAD1, or si-YAP, respectively. (a) The cell viability in each group. (b) The apoptosis of HUVECs in each group. (c) The ROS level in each group. (d) The IL-6 level in each group. (e) The protein expression of VCAM-1 in each group. “∗” means compared with the control group at *P* < 0.05, and “#” means compared with the pcDNA3.1-VGLL4 group at *P* < 0.05. GAPDH was used as an invariant internal control for calculating protein fold changes.

**Table 1:** Primer sequences used in reverse transcription quantitative polymerase chain reaction.

Gene	Primer sequence (5′→3′)
VGLL4	F: AACTGCAACCTCTCGCACTG R: GAGTGGGTGTCGCTGTTGAA
si-TEAD1	F: GGCAUGCCAACCAUUCUUATT
	R: UAAGAAUGGUUGGCAUGCCTT
si-YAP	F: GCAUCUUCGACAGUCUUCUTT
	R: AGAAGACUGUCGAAGAUGCTT
*β*-Actin	F: GATCGATGCCGGTGCTAAGA
	R: TCCTATGGGAGAACGGCAGA

## Data Availability

The datasets used in the present study are available from the authors upon reasonable request.
